# Possible treatment for cutaneous lichen planus: An in vitro anti-inflammatory role of *Angelica* polysaccharide in human keratinocytes HaCaT

This article has been retracted.

**DOI:** 10.1177/2058738418821837

**Published:** 2019-01-08

**Authors:** Jun Wang, Guanzhi Chen, Tongxin Shi, Yingying Wang, Chengfei Guan

**Affiliations:** Department of Dermatology, The Affiliated Hospital of Qingdao University, Qingdao, China

**Keywords:** *Angelica* polysaccharide, cutaneous lichen planus, inflammatory injury, NF-κB pathway, Nrf2/HO-1 pathway, sirtuin 1

## Abstract

Cutaneous lichen planus (CLP) is an autoimmune disease. *Angelica* polysaccharide (AP) has been found to exert immunomodulation activity. In this study, we explored the roles of AP in lipopolysaccharide (LPS)-induced inflammatory injury of human keratinocytes (HaCaT cells), as well as the underlying mechanisms. LPS-induced cell injury was evaluated by alterations of cell viability, apoptosis, and expressions of proteins associated with apoptosis and inflammatory cytokines. Then, the protective effects of AP on LPS-induced cell injury were assessed. The protein expressions of sirtuin 1 (SIRT1) and key kinases in the Nrf2/HO-1 and nuclear factor κB (NF-κB) pathways were measured using western blotting. SIRT1 knockdown and overexpression were used to analyze whether AP affected HaCaT cells through regulating SIRT1. Finally, the possible inhibitory effects of AP on cell injury after LPS treatment were also evaluated. We found that LPS reduced HaCaT cell viability, enhanced apoptosis, and induced release of inflammatory cytokines. AP alleviated LPS-induced HaCaT cell inflammatory injury. The expression of SIRT1 was enhanced after AP treatment. AP activated Nrf2/HO-1 pathway while inhibited NF-κB pathway in HaCaT cells. The protective effects of AP on LPS-induced HaCaT cell injury were reversed by SIRT1 knockdown. Dysregulation of SIRT1 altered the activation of Nrf2/HO-1 and NF-κB pathways in LPS-treated HaCaT cells. Furthermore, AP also exerted inhibitory effects on HaCaT cell injury after LPS stimulation. In conclusion, AP could alleviate LPS-induced inflammatory injury of HaCaT cells through upregulating SIRT1 expression and then activating Nrf2/HO-1 pathway but inactivating NF-κB pathway. This study provided a possible therapeutic strategy for clinical CLP treatments.

## Introduction

Lichen planus (LP) is a common mucocutaneous disease that affects mucous membranes, skin, and appendages of skins (hair and nails).^1^ It was first described in 1869 by a British physician, named Wilson Erasmus, and the estimated prevalence of LP ranged from 0.22% to 5% globally.^2^ LP is rare in children; however, the occurrence of LP in adults with 30–60 years old is relatively high.^3^ As a chronic inflammatory disease, LP is considered to be related to infective, psychogenic, genetic, and autoimmune factors.^4^ Although the exact etiology of LP remains unclear, current literature suggested that autoimmunity is pivotal in LP progression.^5^

Cutaneous lichen planus (CLP) is the most itchy papulosquamous disease, accompanied with characters including polygonal flat-topped, violaceous papules and plaques.^6^ Existing literature are focused on oral lichen planus (OLP);^7,8^ however, investigations about CLP are limited. Currently, a wide range of therapeutic strategies are applied to treat CLP through decreasing the time to lesion resolution, alleviating discomfort, or enhancing life quality. However, the effectiveness and safety of those treatment options have not been proved. More innovative and effective therapeutic strategies are still needed for treatment of CLP.

*Angelica* polysaccharide (AP), the major bioactive component of *Angelica sinensis* (Oliv) Diels, is a β-d-pyranoid polysaccharide with multiple biological activities, such as hematopoiesis, immunomodulation, anti-oxidation, anti-tumor, and radioprotection.^9,10^ For example, Zhang et al.^11^ reported that AP could promote glioma cell apoptosis and inhibit cell growth both in vitro and in vivo. A previous literature has reported that AP possesses immunostimulatory effects on Pacific white shrimps.^12^ Another study also proved that AP could repress the release of pro-inflammatory factors and allergic mediators.^13^ Considering that immune and inflammation are essential in CLP, we hypothesized that AP might affect CLP progression. However, the related literature are limited, which is waiting to be well studied.

Human immortalized keratinocytes (HaCaT cells) maintain full epidermal differentiation capacity.^14^ Lipopolysaccharide (LPS) is a component of the outer membrane of all gram-negative bacteria, and the administration of LPS is frequently applied to investigate inflammation-associated behavior and changes.^15^ In our study, we induced HaCaT cell inflammatory injury using LPS and then explored the possible protective and inhibitory effects of AP on HaCaT cell inflammatory injury in vitro. The underlying molecular mechanisms were also studied. We aimed to discover the potential role of AP in CLP progression.

## Materials and methods

### Cell culture and treatments

Human epidermal keratinocyte cell line, HaCaT, was purchased from the Cell Bank of the Chinese Academy of Sciences (Shanghai, China). HaCaT cells were grown in Dulbecco’s Modified Eagle’s Medium (DMEM; GIBCO, Grand Island, NY, USA) containing 10% fetal bovine serum (FBS; GIBCO) and maintained in a humidified incubator at 37°C with 5% CO_2_. Inflammatory injury of HaCaT cells was induced by incubation in DMEM containing diverse concentrations of LPS (2.5, 5, 10, and 20 μg/mL) for 12 h. AP, purchased from Ci Yuan Biotechnology Co., Ltd., Shanxi (Xian, China), was dissolved in DMEM to generate a 500 μg/mL highly concentrated solution and was further diluted with DMEM to different concentrations (10, 20, 50, 100, and 150 μg/mL). For analyzing possible protective effects of AP on LPS-induced HaCaT cell injury, cells were pre-treated by AP for 24 h prior to LPS stimulation. For analyzing the possible inhibitory effects of AP on HaCaT cell injury after LPS treatment, cells were exposed to LPS for 12 h and then APs were added into the culture medium.

### Cell Counting Kit-8 assay

Viability of HaCaT cells was determined using a Cell Counting Kit-8 (CCK-8) assay (Dojindo Laboratories, Kumamoto, Japan). In brief, transfected or untransfected cells were seeded into 96-well plates with a density of 5 × 10^3^ cells/well. Then, after treatments with LPS and/or AP, 10 μL of CCK-8 solution was added into the culture medium, and these plates were subjected into a humidified incubator for 1 h (37°C, 5% CO_2_). Afterward, measurements of absorbance at 450 nm were carried out using a Microplate Reader (Bio-Rad, Hercules, CA, USA). Cell viability (%) was calculated by average absorbance of LPS (and/or AP) treatment group/average absorbance of control group × 100%.

### FITC annexin V/propidium iodide apoptosis assay

After desired treatments, percentage of apoptotic cells was analyzed using double staining with FITC annexin V and propidium iodide (PI). In brief, after different treatment, transfected or untransfected HaCaT cells were collected after trypsin digestion. Then, after rinsing by phosphate-buffered saline (PBS), cells were resuspended in annexin-binding buffer from a FITC Annexin V/Dead Cell Apoptosis Kit with FITC annexin V and PI for flow cytometry (Invitrogen, Carlsbad, CA, USA). According to the manufacturer’s instructions, cells (100 μL) were stained with 5 μL FITC annexin V and 0.1 μg PI at room temperature for 15 min in the dark. Afterward, stained cells were detected by a FACS can (Beckman Coulter, Fullerton, CA, USA). The percentage of apoptotic cells was analyzed using FlowJo software (Tree Star, San Carlos, CA, USA).

### Transfection and generation of stably transfected cell lines

The full-length human sirtuin 1 (SIRT1) sequences were inserted into pEX-2 to construct pEX-SIRT1. The short-hairpin RNA (shRNA) directed against SIRT1 or a non-targeting sequence was sub-cloned into pGPU6/Neo plasmids (GenePharma, Shanghai, China), and these recombined plasmids were referred to as sh-SIRT1 or sh-NC. Recombined plasmids or empty pEX-2 was transfected into HaCaT cells with the help of the lipofectamine 3000 reagent (Invitrogen) following the manufacturer’s instructions. After transfection, transfected cells were incubated in DMEM supplemented with 0.5 mg/mL G418 (Sigma-Aldrich, St. Louis, MO, USA) to screen stably transfected cells. After approximately 4 weeks, G418-resistant cell clones were established.

### Reverse transcription-quantitative polymerase chain reaction

After desired treatments, total RNA of HaCaT cells was isolated using TRIzol reagent (Invitrogen). Complementary DNA (cDNA) was synthesized by reverse transcription using the PrimeScript™ RT Master Mix (Takara, Dalian, China) according to the manufacturer’s protocol, and 500 ng of RNA acted as template in 10 μL reaction system. The reverse transcription conditions were 15 min at 37°C and 5 s at 85°C, and the products were stored at 4°C. Real-time polymerase chain reaction (PCR) was performed with 7500 Real-Time PCR System (Applied Biosystems, Foster City, CA, USA) using SYBR^®^ Advantage^®^ qPCR Premix, as suggested by the manufacturer. The thermocycling program used was as follows: 30 s at 95°C, followed by 40 cycles of 10 s at 95°C, and 30 s at 60°C. Relative expression of messenger RNAs (mRNAs) was calculated on the basis of the 2-ΔΔCt method,^16^ and β-actin acted as the internal control.

### Preparation of cell lysates and western blot analysis

After desired treatments, HaCaT cells were collected and lysed in radioimmunoprecipitation assay (RIPA) lysis buffer (Beyotime Biotechnology, Shanghai, China) supplemented with protease inhibitors (Beyotime Biotechnology). The proteins in the supernatants of cell lysates were quantified using the BCA™ Protein Assay Kit (Pierce, Appleton, WI, USA). Then, protein samples were loaded into sodium dodecyl sulfate polyacrylamide gel electrophoresis (SDS-PAGE) for separation and transferred to polyvinylidene difluoride (PVDF) membranes. After blocking in 5% non-fat milk, those membranes were incubated with the presence of primary antibody at 4°C overnight, followed by incubation with horseradish peroxidase (HRP)-conjugated secondary antibody (goat anti-rabbit, ab205718; Abcam, Cambridge, UK) for 1 h at room temperature. The primary antibody was against pro-caspase-3 (ab32150), active caspase-3 (ab2302), pro-caspase-9 (ab32539), active caspase-9 (ab2324), interleukin (IL)-1β (ab2105), IL-6 (ab93356), tumor necrosis factor α (TNF-α; ab6671), SIRT1 (ab32441), nuclear factor-erythroid 2-related factor 2 (Nrf2; ab137550), heme oxygenase-1 (HO-1; ab13243), p65 (ab16502), phospho (p)-p65 (ab28856), inhibitor of nuclear factor κB α (IκBα; ab32518), p-IκBα (ab133462), or β-actin (ab8227, Abcam). Protein bands in the PVDF membranes were detected using an ECL Western Blotting Detection Reagent (GE Healthcare, Braunschweig, Germany). The intensities of bands were quantified using the ImageJ software (National Institutes of Health, Bethesda, MA, USA).

### Statistical analysis

All experiments were repeated three times. Results were presented as the mean ± standard error of the mean (SEM). Student’s t test or multiple t tests was used to assess statistical analysis using Graphpad Prism 5 software (GraphPad, San Diego, CA, USA). *P* < 0.05 was considered as a significant difference.

## Results

### LPS-induced HaCaT cell inflammatory injury

HaCaT cells were stimulated with 0, 2.5, 5, 10, or 20 μg/mL LPS for 12 h, and cell viability was measured. Compared with untreated cells, cell viability was significantly decreased by 5 μg/mL (*P* < 0.05), 10 μg/mL (*P* < 0.01), and 20 μg/mL (*P* < 0.001) of LPS stimulation (Figure 1(a)). Since viability of cells stimulated with 10 μg/mL LPS was approximately half of the untreated cells, the 10 μg/mL concentration of LPS was chosen for subsequent experiments. As evidenced in Figure 1(b), percentage of apoptotic cells in the LPS group was markedly higher than that in the control group (*P* < 0.01). The following western blot analysis showed that the expressions of cleaved caspase-3 and cleaved caspase-9 were both notably upregulated by LPS treatments (Figure 1(c)). In addition, we also determined the mRNA and protein expressions of inflammatory cytokines including IL-1β, IL-6, and TNF-α in HaCaT cells after LPS treatment. In Figure 1(d) and (e), the mRNA and protein expressions of these inflammatory cytokines in HaCaT cells were all remarkably upregulated by LPS treatments compared with the control group (*P* < 0.001 in mRNA level). Therefore, we concluded that LPS could induce inflammatory injury of HaCaT cells.

**Figure 1.** LPS-induced inflammatory injury of HaCaT cells. (a) HaCaT cells were stimulated with 0–20 μg/mL LPS for 12 h, and cell viability was determined by CCK-8 assay. Cells were stimulated with 0 (control group) or 10 μg/mL LPS for 12 h. Then, (b) percentage of apoptotic cells, (c) expression of proteins associated with apoptosis, and (d) mRNA and (e) protein expressions of inflammatory cytokines were measured by flow cytometry assay, western blot analysis, RT-qPCR, and Western blot analysis, respectively. Data were presented as the mean ± SEM of three independent experiments. CTRL: control. *P < 0.05; **P < 0.01; ***P < 0.001.

### LPS-induced inflammatory injury was alleviated by AP pre-treatment in HaCaT cells

Next, we aimed to explore the possible protective effects of AP on LPS-induced inflammatory injury of HaCaT cells. First of all, cells were stimulated with diverse concentrations of AP (0, 10, 20, 50, 100, and 150 μg/mL) to explore the adequate dosage. In Figure 2(a), there were no significant effects of AP on cell viability when the concentration of AP was 10, 20, 50, or 100 μg/mL. However, 150 μg/mL AP could significantly reduce cell viability compared with untreated cells (*P* < 0.05). Hence, the concentration of AP in subsequent experiments was 100 μg/mL. Then, cells were treated with LPS or AP plus LPS, followed by measurements of cell viability, apoptosis, and expressions of proteins associated with apoptosis and inflammatory cytokines. Interestingly, those LPS-induced alterations were all significantly attenuated by AP pre-treatment, as compared to the LPS group (*P* < 0.05 or *P* < 0.01; Figure 2(b)–(f)). Results collectively illustrated that AP pre-treatment could alleviate LPS-induced inflammatory injury of HaCaT cells.

**Figure 2.** LPS-induced inflammatory injury of HaCaT cells was alleviated by *Angelica* polysaccharide (AP) pre-treatments. (a) HaCaT cells were stimulated with 0–150 μg/mL AP for 48 h, and cell viability was determined by CCK-8 assay. Cells were stimulated with 10 μg/mL LPS or 100 μg/mL AP plus 10 μg/mL LPS. Non-treated cells acted as control. Then, (b) cell viability, (c) percentage of apoptotic cells, (d) expression of proteins associated with apoptosis, and (e) mRNA and (f) protein expressions of inflammatory cytokines were measured by CCK-8 assay, flow cytometry assay, western blot analysis, RT-qPCR, and Western blot analysis, respectively. Data were presented as the mean ± SEM of three independent experiments. CTRL: control. *P < 0.05; **P < 0.01; ***P < 0.001.

### AP-upregulated protein expression of SIRT1 in HaCaT cells

We next explored the possible regulatory mechanism of AP in LPS-treated cells. Accordingly, the protein expressions of SIRT1 in cells treated with LPS or AP plus LPS were assessed. In Figure 3, SIRT1 protein expression was dramatically downregulated by LPS treatments compared with the control group (*P* < 0.01). However, the effects of LPS on SIRT1 expression were notably reversed by AP pre-treatment relative to the LPS group (*P* < 0.001). Those results suggested that SIRT1 might be involved in the modulation of AP in LPS-treated HaCaT cells.

**Figure 3.** *Angelica* polysaccharide (AP) upregulated SIRT1 expression in HaCaT cells. HaCaT cells were stimulated with 10 μg/mL LPS or 100 μg/mL AP plus 10 μg/mL LPS. Non-treated cells acted as control. Then, SIRT1 protein expression was assessed by western blot analysis. Data were presented as the mean ± SEM of three independent experiments. CTRL: control. **P < 0.01; ***P < 0.001.

### AP activated the Nrf2/HO-1 pathway while inactivated the NF-κB pathway in HaCaT cells

The involvements of the Nrf2/HO-1 and NF-κB pathways in the modulation of AP in LPS-treated HaCaT cells were also studied. As compared to the control group, LPS significantly upregulated the expressions of Nrf2 and HO-1 (*P* < 0.05 or *P* < 0.001; Figure 4(a)) and remarkably increased the phosphorylated levels of p65 and IκBα (both *P* < 0.001; Figure 4(b)). Meanwhile, LPS-induced upregulations of Nrf2 and HO-1 were further upregulated by AP pre-treatment relative to the LPS group (both *P* < 0.01). Conversely, LPS-induced increases of p-p65 and p-IκBα were significantly abrogated by AP pre-treatment relative to the LPS group (*P* < 0.01 or *P* < 0.001). Collectively, we concluded that AP could activate the Nrf2/HO-1 pathway while inactivate the NF-κB pathway in HaCaT cells.

**Figure 4.** *Angelica* polysaccharide (AP) activated the Nrf2/HO-1 pathway while inhibited the NF-κB pathway in HaCaT cells. HaCaT cells were stimulated with 10 μg/mL LPS or 100 μg/mL AP plus 10 μg/mL LPS. Non-treated cells acted as control. Then, expressions of key kinases in (a) the Nrf2/HO-1 pathway and (b) the NF-κB pathway were evaluated by western blot analysis. Data were presented as the mean ± SEM of three independent experiments. CTRL: control; t-: total; p-: phospho-. *P < 0.05; **P < 0.01; ***P < 0.001.

### AP affected LPS-treated HaCaT cells through upregulating SIRT1 expression

Subsequent experiments were performed to ascertain whether AP affected LPS-treated HaCaT cells through upregulating SIRT1 expression. First of all, recombined plasmids were stably transfected into HaCaT cells, and the expression of SIRT1 was measured. Western blot result in Figure 5(a) shows that SIRT1 expression in the pEX-SIRT1 group was significantly higher than that in the pEX group (*P* < 0.001), and SIRT1 expression in the sh-SIRT1 group was markedly lower than that in the sh-NC group (*P* < 0.01). This result indicated that SIRT1 expression could be successfully dysregulated by stable transfection. Then, transfected and untransfected cells were treated with LPS or AP plus LPS, followed by measurements of inflammatory injury. As can be evidenced from Figure 5(b)–(f), effects of AP on LPS-treated cells were all markedly abrogated by SIRT1 knockdown, as compared to the AP + LPS + sh-NC group (*P* < 0.05 or *P* < 0.01). The above-mentioned data proved that the upregulation of SIRT1 expression might be a reason for the protective effects of AP on HaCaT cells.

**Figure 5.** Effects of *Angelica* polysaccharide (AP) pre-treatments on HaCaT cell were reversed by SIRT1 knockdown. (a) HaCaT cells were transfected with pEX-2, pEX-SIRT1, sh-NC, or sh-SIRT1 and expression of SIRT1 was measured by western blot analysis. Transfected and untransfected cells were stimulated with 10 μg/mL LPS or 100 μg/mL AP plus 10 μg/mL LPS. Non-treated cells acted as control. Then, (b) cell viability, (c) percentage of apoptotic cells, (d) expression of proteins associated with apoptosis, and (e) mRNA and (f) protein expressions of inflammatory cytokines were measured by CCK-8 assay, flow cytometry assay, western blot analysis, RT-qPCR, and western blot analysis, respectively. Data were presented as the mean ± SEM of three independent experiments. CTRL: control. *P < 0.05; **P < 0.01; ***P < 0.001.

### SIRT1 overexpression activated the Nrf2/HO-1 pathway while inhibited the NF-κB pathways in LPS-treated HaCaT cells

We also explored the effects of dysregulated SIRT1 on the Nrf2/HO-1 and NF-κB pathways. Results in Figure 6(a) show that LPS-induced upregulations of Nrf2 and HO-1 were further upregulated by SIRT1 overexpression (both *P* < 0.001) while were reversed by SIRT1 knockdown (both *P* < 0.001) as compared to respective controls. Oppositely, LPS-induced increases in p-p65 and p-IκBα were significantly reversed by SIRT1 overexpression (*P* < 0.01 or *P* < 0.001) while were further increased by SIRT1 knockdown (*P* < 0.05 or *P* < 0.01; Figure 6(b)). Those results indicated that SIRT1 dysregulation could affect the activation of the Nrf2/HO-1 and NF-κB pathways in LPS-treated HaCaT cells.

**Figure 6.** Dysregulated SIRT1 affected the Nrf2/HO-1 and the NF-κB pathways in HaCaT cells. Transfected and untransfected HaCaT cells were stimulated with 10 μg/mL LPS for 12 h. Non-treated cells acted as control. Then, expressions of key kinases in (a) the Nrf2/HO-1 pathway and (b) the NF-κB pathway were evaluated by western blot analysis. Data were presented as the mean ± SEM of three independent experiments. CTRL: control; t-: total; p-: phospho-. *P < 0.05; **P < 0.01; ***P < 0.001.

### AP post-treatment also attenuated the LPS-induced HaCaT cell inflammatory injury and upregulated the expression of SIRT1

Finally, we also assessed the effects of AP on HaCaT injury after LPS stimulation. Results in Figure 7(a) and (b) show that AP post-treatment also significantly alleviated the LPS-induced cell viability inhibition and cell apoptosis (*P* < 0.05). The protein expressions of cleaved-caspase 3 and cleaved-caspase 9 were both decreased in LPS-treated HaCaT cells after AP post-treatment (Figure 7(c)). Moreover, Figure 7(d) presents that compared to LPS group, the protein expressions of IL-1β, IL-6, and TNF-α in HaCaT cells were all reduced after LPS + AP post-treatment. Figure 7(e) displays that AP post-treatment also remarkably reversed the LPS-induced downregulation of SITR1 in HaCaT cells (*P* < 0.01). Taken together, these above results suggested that AP also could attenuate the LPS-induced HaCaT cell inflammatory injury and upregulate the expression of SIRT1.

**Figure 7.** AP post-treatment also attenuated the LPS-induced HaCaT cell inflammatory injury and upregulated the expression of SIRT1. HaCaT cells were stimulated with 10 μg/mL LPS for 12 h and then exposed to 100 μg/mL AP for 24 h. Non-treated cells acted as control. Then, (a) cell viability, (b) percentage of apoptotic cells, (c) expression of proteins associated with apoptosis, (d) expression of inflammatory cytokines, and (e) expression of SIRT1 were measured by CCK-8 assay, flow cytometry assay, and western blotting, respectively. Data were presented as the mean ± SEM of three independent experiments. CTRL: control. *P < 0.05; **P < 0.01.

## Discussion

Patients with CLP may feel embarrassed due to the intense itch in some cases. In addition, the lesions due to CLP may lead to long-standing residual hyperpigmentation.^17,18^ Thus, it is an urgent need to explore effective therapies for CLP. CLP appears to be an autoimmune disease; an autoimmune disease is a disorder by which the body’s own immune system attacks healthy cells, and the inflammation is the common symptom of an autoimmune disease.^19^ Therefore, we focused on inflammatory injury of keratinocytes to explore the possible therapeutic drug for CLP. LPS is a potent inflammatory stimulus. Results in our study showed that HaCaT cell viability was reduced and percentage of apoptotic cells was enhanced under LPS stimulation. Activation of caspases is closely associated with cell apoptosis. Activated caspase-9 can subsequently induce activation of caspase-3, regulating enhanced cell apoptosis.^20^ The alteration of active caspase-9 and caspase-3 after LPS treatments consolidated that LPS induced cell apoptosis. Moreover, release of pro-inflammatory cytokines including IL-1β, IL-6, and TNF-α was elevated by LPS treatments. All the results illustrated that inflammatory injury of HaCaT cells was successfully induced by LPS.

Previous studies have proved the anti-inflammatory and immunoregulatory functions of AP.^9,10^ Thus, we hypothesized that AP may attenuate inflammatory injury of HaCaT cells. Unsurprisingly, under pre-treatment of 100 μg/mL AP, LPS-induced reduction in cell viability, enhancements of cell apoptosis, and elevated release of inflammatory cytokines were all alleviated. The results of our study were consistent with previous literature. For example, the literature by Zhuang et al.^21^ showed that H_2_O_2_-induced injury of chondrocytes was reduced by AP. Lei et al.^22^ also proved that oxidative stress–induced neuronal cell injury was alleviated by AP. In addition, Wang and Wu^23^ found that AP could inhibit inflammation in both HepG2 cells and rats with anemia of chronic disease. Moreover, considering that we also found that 150 μg/mL AP treatment significantly inhibited the viability of HaCaT cells, which suggested that AP in high concentration might have some adverse effects and biological limitation. Further research works are still needed to analyze the dosage selection of AP on CLP treatment.

SIRTs are conserved NAD^+^-dependent deacetylases and ADP-ribosyltransferases that participate in diverse cellular processes, such as DNA repair, gene silencing, and metabolic regulation.^24^ SIRT1 is a longevity protein which is required for long-term growth of human mesenchymal stem cells.^25^ Moreover, it is involved in multiple biological processes, including cell apoptosis, senescence, metabolism, and inflammation.^26^ Dal Farra and Domloge^27^ reported that SIRT1 was expressed in cultured HaCaT cells and its level was closely related to stress and aging. Kim^28^ proved that SIRT1 played critical roles in the protective effects of garlic, a flavoring agent, on UVB-exposed HaCaT human keratinocytes. SIRT1 has also been demonstrated to be involved in the regulation of circadian oscillation of keratinocytes, including HaCaT cells.^29^ In addition, Wang et al.^30^ reported that AP can activate SIRT1-AMPK signaling cascade. Therefore, we hypothesized that there might be a relationship between AP and SIRT1 expression in HaCaT cells. Western blot results showed that LPS-induced downregulation of SIRT1 expression was reversed by AP pre-treatment. Moreover, effects of AP pre-treatment on cell viability, apoptosis, and release of inflammatory cytokines in LPS-treated HaCaT cells were significantly reversed by SIRT1 knockdown, reinforcing that AP exerted protective effects on HaCaT cell injury through upregulating SIRT1 expression.

Nrf2 has been reported to protect cells against inflammatory injuries via regulation of NADPH, glutathione peroxidase, HO-1, and anti-oxidant genes.^31^ It can regulate gene expression and inflammation in keratinocytes.^32^ In addition, the Nrf2/HO-1 signaling pathway plays a major role in anti-inflammatory functions.^31^ The NF-κB pathway is reported as a critical regulator of proliferation, survival, apoptosis, and inflammation.^33^ Normally, p65 was bound to IκBα and located in cytoplasm. LPS can induce phosphorylation of IκBα, followed by dissociation between p65 and IκBα as well as phosphorylation of p65. Then, p-p65 translocates into the nucleus and then induces expression of inflammatory factors.^34–36^ Therefore, we explored the involvements of the Nrf2/HO-1 and NF-κB pathways in AP-associated regulations. Results showed that AP could activate the Nrf2/HO-1 pathway while inhibit the NF-κB pathway. Moreover, SIRT1 overexpression could activate the Nrf2/HO-1 pathway but inhibit the NF-κB pathway, indicating that dysregulated SIRT1 could affect the activation of these two pathways. These results collectively illustrated that AP could affect the Nrf2/HO-1 and NF-κB pathways through upregulating SIRT1.

Finally, we also assessed the effects of AP on HaCaT injury after LPS stimulation and found that AP also could exert inhibitory effects on HaCaT cell injury after LPS stimulation and upregulate the expression of SIRT1. Taken together, the findings of our research indicated that both AP pre-treatment or post-treatment could alleviate LPS-induced inflammatory injury of HaCaT cells through upregulating SIRT1 expression. In addition, AP could activate the Nrf2/HO-1 pathway but inhibit the NF-κB pathway through SIRT1-mediated regulations. This study established the foundation for deep investigations of AP function and it provided possible therapeutic strategies for clinical CLP treatments.

Our study is a very simple experimental research about the effects of AP on potential cell-based model of CLP. Until now, there is no information available about the experimental animal model of CLP. Some reports indicated that LPS-induced HaCaT cell damage could simulate LP, especially OLP. For example, Wang et al. indicated that total glucosides of paeony (TGP) inhibited the LPS-induced production of inflammatory cytokines in OLP by suppressing NF-κB signaling pathway.^37^ Another report proved that miR-125b was involved in the LPS-induced keratinocyte HaCaT cell proliferation inhibition and apoptosis in OLP via targeting MP-2 expression through PI3K/AKT/mTOR pathway.^38^ More research works or in vivo animal experiments are needed to further verify the anti-inflammatory effect of AP on CLP in the future.
